The article "A case–control study of drinking beverages and the risk of multiple sclerosis in Iran" was published in 2023. Journal: J Health Popul Nutr.

# A case–control study of drinking beverages and the risk of multiple sclerosis in Iran

**DOI:** 10.1186/s41043-023-00364-8

**Published:** 2023-03-23

**Authors:** Maryam Dastoorpoor, Seyed Massood Nabavi, Nastaran Majdinasab, Ahmad Zare Javid, Kambiz Ahmadi Angali, Maryam Seyedtabib

**Affiliations:** 1 Department of Biostatistics and Epidemiology, Musculoskeletal Rehabilitation Research Center, Ahvaz Jundishapur University of Medical Sciences, Ahvaz, Iran; 2 Department of Regenerative Biomedicine, Royan Institute for Stem Cell Biology and Technology, ACCR, Tehran, Iran; 3 Department of Brain and Cognition, Royan Institute for Stem Cell Biology and Technology, ACCR, Tehran, Iran; 4 Department of Neurology, Musculoskeletal Rehabilitation Research Center, Ahvaz Jundishapur University of Medical Sciences, Ahvaz, Iran; 5 Department of Nutritional Sciences, School of Allied Medical Sciences, Nutrition, and Metabolic Disease Research Center, Ahvaz Jundishapur University of Medical Sciences, Ahvaz, Iran; 6 Department of Biostatistics and Epidemiology, School of Public Health, Ahvaz Jundishapur University of Medical Sciences, Ahvaz, Iran

**Keywords:** Multiple sclerosis, Beverages, Carbonated beverages, Coffee, Black tea, Green tea

## Abstract

**Background:**

There is no study in the world on the relationship between consuming black and green tea as beverages containing polyphenols and the risk of MS. This study aimed to determine the association between the consumption of green and black tea, coffee, non-alcoholic beer, milk, fruit juices and carbonated beverages with the risk of MS.

**Methods and materials:**

This case–control study was performed on 150 patients with MS and 300 healthy individuals as a control group among patients who were referred to the ophthalmology ward of a referral hospital in Ahvaz with the groups matching for age. The data collection tool was a researcher-made questionnaire including demographic information and beverage consumption. Analysis was performed using univariate and multiple logistic regression models.

**Results:**

The mean age of patients at the time of diagnosis was 38.55 ± 8.88 years. The results showed that drinking milk (OR = 5.46), natural juice (OR = 2.49), and carbonated beverages (OR = 16.17) were associated with an increased chance of developing MS. However, drinking non-alcoholic beer (OR = 0.48), black tea (OR = 0.20), green tea (OR = 0.29) and coffee (OR = 0.07) were associated with a reduced chance of developing MS.

**Conclusion:**

The results show that drinking black and green tea, non-alcoholic beer, and coffee are associated with a decrease in the chance of developing MS. The results of this study can be used to design interventional research and to change people's lifestyles to prevent MS.

## Introduction

Multiple sclerosis (MS) is a disease of the nervous system that gradually destroys nerve fibers as a result of the progression of the disease. This is probably the cause of the disabilities occurring among these patients [1–4]. More than two million individuals worldwide suffer from MS [5]. More individuals in Asia and the Middle East have MS than in the east and southeast [6]. Colder countries have the highest prevalence of MS worldwide [7]. The average global prevalence of the disease rose from approximately 29 per 100,000 in 2013 to 44 per 100,000 in 2020 [8]. The prevalence of the disease in Iran has increased dramatically in the last twenty years [9, 10]. Khuzestan Province (southwest Iran) has been reported as a dangerous region with a prevalence and average annual incidence of around 58 and 4.35 per 100,000 individuals from 2006 to 2019, respectively [11].

In most cases, MS symptoms occur between the ages of 20, and 40 [4, 12]. The underlying cause of MS is yet to be known [13]. However, various studies have shown that different factors increase or decrease the risk of developing MS, including being female, genetics, environment, climate, smoking, high-fat diet, and coffee consumption [14–17]. Some evidence suggests that genetic factors predispose some people to MS [18]. However, genetic predisposition is only part of the explanation of the mechanism; other factors seem to affect the onset of the disease in susceptible individuals [9]. Controlling the genetic factor is basically beyond human reach. However, attention to the environmental factors, which have recently played a very important role in the incidence, recurrence, and treatment of the disease, can be largely controlled by humans [19]. Some individual behavior factors such as smoking, smoking pipe, and hookah, also the consumption of drinks, such as coffee, alcohol, and polyphenol beverages are studied to determine their role in developing MS [20, 21]. One of the possible environmental factors that can play a protective role in some non-communicable diseases is coffee. Coffee contains more than a thousand biologically active compounds that contain caffeine and is a stimulant of the central nervous system in animal and human beings [22]. Caffeine has a protective role in Alzheimer's disease in animal models. Studies also show that caffeine use reduces cerebral inflammation and intracranial hemorrhage in animal models with MS [23–25]. In a study by Hedström et al. [26], the results showed that very high coffee consumption in the animal model reduces the risk of multiple sclerosis. Few epidemiological studies have been performed on the effect of coffee on humans in developing MS. Regarding the inverse association between coffee and the risk of MS in humans, several studies have been reported with conflicting results. Some studies reported no evidence [25, 27–29]. A study by Jahromi et al. [30] examined seven possible dietary patterns for MS. Their results show that the first dietary pattern (including the traditional dietary pattern: increase in consumption of low-fat dairy products, red meat, vegetable oils, onions, whole grains, soybeans, refined grains, organic meats, coffee, beans, and butter) have adverse effects on the risk of MS. Meanwhile, the risk of MS was very high in those on a high-fat diet and animal products (potatoes, meat, sugars, hydrogenated and low-fat fats, spices, and skinless chicken) [30]. The study by D’hooghe et al. [17] aimed at investigating the role of alcohol, coffee, fish, and smoking on the progression of disability, recurrence, and onset of MS attacks, showed that people who have recently developed MS have a risk of progression. Early disability is reduced in alcohol, wine, and coffee consumers compared to those who have never consumed these substances.

Studies have shown that, due to their multiple protective effects, polyphenols have antioxidant, anti-inflammatory, anti-aging, cardiovascular protective activity, and neuroprotein effects. Because many polyphenols are widely distributed in plant cells, they are used almost daily in the diet (including tea in the Iranian culture). Currently, a few findings suggest that resveratrol, as a polyphenol, is a promising weapon for the prevention and treatment of cancer and many other diseases. Many studies have also shown that polyphenols have biological and biochemical protective effects on the heart, blood circulation, brain, and age-related diseases [31].

There is no study in the world on the relationship between consuming black and green tea as beverages containing polyphenols and the risk of MS. MS is on the rise and there are not enough studies on the role of environmental factors affecting it. Therefore, this study aimed to determine the relationship between the consumption of green and black tea, coffee, non-alcoholic beer, milk, natural and packaged fruit juices, and carbonated beverages and the risk of MS in a case–control study.

## Methods

This research was a hospital-based case–control study in which the case group includes patients with MS. The control group was patients referring to the ophthalmology ward of Imam Khomeini hospital in Khuzestan province as a referral hospital. The control group was matched for age (at intervals of 5).

### Case group

The Khuzestan Province MS Association, as the only MS center in the neurology department of a referral hospital in Ahvaz, was used to register MS patients. Eligibility criteria included: Being 15 to 50 years old, being definitively diagnosed with MS by at least one neurologist (using McDonald criteria in the initial stage and final confirmation of the diagnosis by MRI), and living in eight areas of Ahvaz Municipality at the time of diagnosis. Exclusion criteria include: Unwillingness to cooperate, inability to talk, and a decrease in the level of consciousness.

### Control group

Among the types of controls available in case–control studies (friends, family, neighbors, hospital, random sample of a population), hospital controls were used in the ophthalmology ward of a referral hospital in Ahvaz, Iran. Therefore, only living individuals who did not have MS and lived in 8 districts of Ahvaz were considered as controls and were grouped in terms of age. The reason for selecting the control group from the eye department was the lack of relationship between the disease in the control group and the exposure. Based on similar studies, three factors of age, gender, and education level were important confounders. This research adjusted age with enlivening matching, and gender and education levels were modified in the analysis stage with the logistic model.

### Sample size

According to a similar study based on coffee consumption in two groups and taking into account the 95% confidence level and 80% test power, the sample size (n2 = k.n1) was estimated at 150 for patients [32, 33]. Because the ratio of control to the case was taken as *k* = 2, 300 hospital controls in the age group of 15–50 years were included. However, after completing the questionnaires the participants and deleting the questionnaires at least 20% of the questions had no answer, and the sample size in the two groups of patients and controls reached 146 and 277, respectively. The response rate was 94.0% (Fig. 1).

**Fig. 1:** Flowchart of the study

Data collection tools in this study consisted of a checklist including two parts: (a) Demographic characteristics (age, sex, marital status, and level of education), (b) Consumption of beverages including Milk, natural juices, packaged juices, non-alcoholic beer, black tea, green tea, coffee, and soft drinks. Regarding categories of consumption for each beverage, all beverages except the two black and green tea are divided into two categories (with/without) consumption. According to the high consumption of tea in Iran, two cut points were considered to classify the consumption of black (< 500 g/day) and green (< 16 g/day) tea using the ROC curve.

### Statistical analysis

In the descriptive statistics section, the mean, frequency, and standard deviation were used. To estimate the odds ratio and 95% confidence interval, univariate, and multiple logistic regression models were performed. SPSS software (version 16) was used to analyze the data. The significance level is considered less than 0.05.

## Results

The mean (SD) age of participants in the case group was 38.55 (8.88), and for those in the control group, it was 37.24 (9.47). Table 1 shows that around 20% of participants in the case groups were male, whereas 42% were male in the control group. The percentages of participants with an academic education for the case and control groups were 54.8% and 34.7%, respectively. Sixty percent and 20.6% of participants in the case and control group, respectively, had had a history of milk consumption during adolescence. This result for coffee consumption in the case and control group was 24.7% and 43.0%, respectively. Others results are shown in Table 1.

**Table 1:** Frequency distribution of demographic and drinking beverages variables in the case and control group

Participant Characteristics	Level	Case = 146		Control = 277	
		*N*	%	*N*	%
Gender	Female	117	80.10	162	58.50
	Male	29	19.90	115	41.50
Marital status	Single	38	26.00	68	24.50
	Married	100	68.50	168	60.60
	Divorced/widow	8	5.50	41	14.80
Education	Less than high school	19	13.10	78	28.10
	High school	47	32.20	103	37.20
	University	80	54.80	96	34.70
Milk (g/day)	0	58	39.70	220	79.40
	> 0	88	60.30	57	20.6
Natural juice (g/day)	0	59	40.40	184	66.40
	> 0	87	59.60	93	33.60
Juice packet (g/day)	0	74	50.70	194	70.00
	> 0	72	49.40	83	30.00
Non-alcoholic beer (g/day)	0	98	67.10	178	64.30
	> 0	48	32.90	99	35.70
Black tea (g/day)	< 500	107	73.70	109	39.40
	≥ 500	39	24.70	168	60.60
Green tea (g/day)	< 16	132	90.40	223	80.50
	≥ 16	14	9.60	54	19.50
Coffee (g/day)	0	110	75.30	158	57.00
	> 0	36	24.70	119	43.00
Carbonated beverages (g/day)	0	42	28.80	155	56.00
	> 0	104	71.20	122	44.00

The adjusted estimates of odds ratios (ORs) for different factors for MS are shown in Table 2. The results of multiple logistic regression models showed that the ORs of MS relating to the gender and university level of education was 0.317 [0.161–0.624] and 3.329 [1.484–7.467] respectively. In other words, the risk of developing MS in females was 3.2 times higher than in males. Also, the participants with a university education had more likely to have MS than the group with less than high school. All drinks, except Juice packets (OR = 1.533 [0.81–2.91], have significant relation with MS. Of these, more intake of carbonated beverages ((> 0 g/day), OR = 16.17 [5.99–43.61]), milk (> 0 g/day), OR = 5.46 [2.84–10.49] and natural juice ((> 0 g/day), OR = 2.48 [1.31–4.71]) were risk factors and more intake of coffee ((> 0 g/day), OR = 0.07 [0.03–0.18]), black tea ((≥ 500 g/day), OR = 0.20 [0.11–0.37]), green tea ((≥ 16 g/day), OR = 0.29[0.13–0.64]), and drinking non-alcoholic beer ((> 0 g/day), OR = 0.48 [0.24–0.96]) had a positive relation against MS. Based on the results, the participants who had no coffee consuming experience are 14.5 times more likely to develop MS than those who drink coffee.

**Table 2:** The important risk factors for multiple sclerosis (univariate and multivariate logistic regression models)

Variable	Crude OR				Adjusted OR			
	OR	95% CI		*P*-value	OR	95% CI		*P*-value
		Lower	Upper			Lower	Upper	
Gender (Ref: female)	–	–	–	–	–	–	–	–
Male	0.349	0.218	0.560	< 0.001	0.317	0.161	0.624	0.001
Marital status (Ref: single)	–	–	–	–	–	–	–	–
Married	1.056	0.667	1.701	0.791	1.383	0.704	2.715	0.347
Divorced/widow	0.349	0.148	0.821	0.016	0.482	0.153	1.521	0.213
Education (Ref: less than high school)	–	–	–	–	–	–	–	–
High school	1.873	1.019	3.443	0.043	1.815	0.788	4.183	0.162
University	3.421	1.910	6.126	< 0.001	3.329	1.484	7.467	0.004
Milk (Ref: 0 g/day)	–	–	–	–	–	–	–	–
> 0	5.856	3.767	9.104	< 0.001	5.458	2.841	10.487	< 0.001
Natural juice (Ref: 0 g/day)	–	–	–	–	–	–	–	–
> 0	2.917	1.928	4.414	< 0.001	2.485	1.312	4.707	0.005
Juice packet (Ref: 0 g/day)	–	–	–	–	–	–	–	–
> 0	2.274	1.503	3.440	< 0.001	1.533	0.809	2.906	0.190
Non-alcoholic beer (Ref: 0 g/day)	–	–	––	–	–	–	–	–
> 0	0.881	0.567	1.345	0.557	0.481	0.241	0.960	0.038
Black tea (Ref: < 500 g/day)	–	–	–	–	–	–	–	–
≥ 500	0.236	0.152	0.367	< 0.001	0.199	0.106	0.371	< 0.001
Green tea (Ref: < 16 g/day)	–	–	–	–	–	–	–	–
≥ 16	0.438	0.234	0.819	0.010	0.289	0.130	0.642	0.002
Coffee (Ref: 0 g/day)	–	–	–	–	–	–	–	–
> 0	0.435	0.278	0.678	< 0.001	0.067	0.025	0.182	< 0.001
Carbonated beverages (Ref: 0 g/day)	–	–	–	–	–	–	–	–
> 0	3.146	2.047	4.835	< 0.001	16.168	5.994	43.613	< 0.001

*CI* confidence interval, *OR* odds ratio, *Ref* reference level

## Discussion

This study aimed to determine the association between the consumption of green and black tea, coffee, non-alcoholic beer, milk, fruit juices and carbonated beverages with the risk of MS. Our results showed that drinking carbonated beverages significantly increases the chances of developing MS by 16 times. The results of a meta-analysis study by Narain et al. [34] showed that increasing the consumption of carbonated sugary drinks increases cardiovascular problems and stroke. A cross-sectional study by Conlay et al. [35] showed that there is a significant relationship between increasing the consumption of any combination of sugary drinks (except diet drinks) and increasing the chance of developing arthritis in the age group of 20 to 30 years.

Our results showed that milk significantly increases the chances of developing MS by five times. This is inconsistent with a case–control study by Dehghan and Ghaedi-Heidari [36], which showed that the use of cow's milk in infancy and avoiding plant-based diets reduces the chances of developing MS. Another study by Harirchian et al. showed that drinking cow milk before puberty triggers an autoimmune process and increases the risk of MS in adulthood [37]. Our results showed that the consumption of natural fruit juice significantly increases the chances of developing MS by 2.5 times. A cross-sectional study by DeChristopher et al. [38] found that consuming any combination of sugary drinks, fruit drinks, and apple juice was significantly associated with coronary artery problems in adults. Adults who drank these drinks five times a week were 2.8 times more likely to develop coronary artery disease than those who drank three times a week. Researchers in the study acknowledged that sugary drinks, fruit drinks, and apple juice may contribute to cardiovascular disease, chronic respiratory disease, and autoimmune arthritis. This is probably due to the high ratio of fructose to glucose in these drinks [38].

Our results also showed that drinking coffee, black and green tea, and non-alcoholic beer significantly reduce the risk of MS and have protective properties. A study by Hedström et al. [26] in two independent case–control studies showed that excessive consumption of coffee reduces the risk of MS. Also, in a cross-sectional study by D’hooghe et al. [17] on 1372 patients with MS, the results showed that drinking coffee, alcohol, and eating fish have an inverse relationship with the development of disability in MS.

In addition, in a systematic review and meta-analysis by Herden and Weissert [39], the results showed that drinking coffee, especially caffeine, if consumed in relatively high doses, has a preventive role in causing several neurodegenerative diseases. There was a significant relationship between drinking coffee and the risk of MS and Parkinson's disease; drinking coffee showed a protective effect [39]. A study with a 21-year follow-up study also found that drinking 3–5 cups of coffee on average per day significantly reduces the risk of Alzheimer's disease [35, 40, 41].

Coffee, black tea, and green tea contain caffeine. Caffeine (1, 3, 7-trimethylxanthine) acts as a psychological stimulant in the central nervous system (CNS). The stimulant effects of caffeine are due to its ability to reduce adenosine transport in different areas of the brain [42]. The underlying mechanism of the neuroprotective effect of caffeine is not fully understood, however, a beneficial effect can be observed in various organisms and conditions of chronic and autoimmune diseases [39]. Some studies have also shown that black and green tea and coffee contain high levels of polyphenols and other phytochemicals that have anti-inflammatory characteristics, suppress pro-inflammatory cytokines, reduce neuronal damage and protect the nervous system [39, 43, 44].

Our results also showed that the chance of developing MS in women is 3.2 times higher than in men, which is consistent with a review study by Olsson et al. [45] who showed that the prevalence of MS in women is higher than in men [45, 46].

Women with MS show more inflammatory lesions on MRI than men, and women also have a higher age of onset [47, 48]. Studies have shown that MS affects women three times more often than men [49–51]. It has been assumed that hormonal changes such as estrogen, progesterone, testosterone, etc. may be partly responsible for this [45, 46]. The results also showed that people with a college education 3.36 times are more likely to develop MS than those with a high school education. This is inconsistent with a study by Magyari et al. [52], Bjørnevik et al. [53], Riise et al. [54], and Briggs et al. [55].

One of the strengths of our study is that it seems that this study was the first that examined the relationship between drinking tea, non-alcoholic beer, milk, and fruit juice with a chance of developing MS. Also, patients were selected from the MS Association as the only patient registration center in Ahvaz. One of the limitations of the study is that due to the nature of the study, which is a case–control study, there is a possibility of memory bias; Individuals may not recall their past experiences properly. Therefore, it is suggested that future research focuses on case–control (nested) or case–control (case-group) research, as in these two types of studies, it is not possible to create a recall bias.

## Conclusion

The results of this research showed that drinking coffee, black and green tea, and non-alcoholic beer has protective properties and reduce the chances of developing MS. On the other hand, consuming carbonated beverages, milk, and fruit juices except packaged fruit juice reduces the chances of developing MS. The results of this study can be used to design interventional research and to change people's lifestyles to prevent MS.

## Data Availability

The datasets generated and/or analyzed during the current study are not publicly available due to the necessity to ensure patient confidentiality policies but are available from the corresponding author on reasonable request.
